# Evaluation of Emergency Intelligence Capability of Major Public Health Events in Probabilistic Uncertain Language Environment

**DOI:** 10.1155/2022/1302598

**Published:** 2022-02-26

**Authors:** Yaxu Yang, Zixue Guo

**Affiliations:** School of Management, Hebei University, Baoding 071000, China

## Abstract

Emergency intelligence capability is an important index reflecting the intelligence level of emergency management. The accuracy of emergency intelligence capability evaluation is related to the scientific nature of emergency decision-making. By analyzing the operation process and mechanism of the emergency intelligence system for major public health events, this paper establishes the evaluation index system of the emergency intelligence capability. By using the decision method of VIKOR and considering the preference of experts in the evaluation process, this paper proposes the evaluation model based on the probabilistic uncertain language environment. The use of probabilistic uncertain linguistic term set (PULTS) to describe the uncertain information is helpful to improve the scientific and accuracy of emergency rescue decision-making of major public health events and then realize the organic unity of emergency information and scientific decision-making of public health events.

## 1. Introduction

Major public health event is a kind of public crisis, which has the characteristics of unpredictability, abruptness, and particularity. Establishing and improving the evaluation system of emergency intelligence capability is the basis of improving the efficiency of dealing with major public health event. There was a variety of major public health events endangering human beings, including plague, smallpox, cholera, leprosy, diphtheria, syphilis, typhus, malaria, rabies, tuberculosis, and dozens of other diseases. They brought varying degrees of harm to human beings, with plague and smallpox being the most important. In recent years, major public health events have occurred frequently. The outbreak of SARS in 2003, the outbreak of Ebola virus in West Africa, and the raging COVID-19 pandemic have posed serious threats to people's lives and health as well as economic and social development. According to the latest real-time statistics from WHO by December 2021, 265.19 million COVID-19 cases had been confirmed worldwide, with more than 5.25 million deaths, causing heavy casualties and huge economic losses. China attaches great importance to the prevention and control of major public health incident, and the communist party of China in the 19th the fifth plenary session proposed “resolve major risk systems and mechanisms to prevent constantly improved, markedly enhance its capability of public emergency response” of the social development main goal and set up with infectious disease and public health emergency monitoring as the core of information system of disease prevention and control in China. At present, the Chinese government and all sectors of society pay great attention to the construction of emergency intelligence capability evaluation system. However, due to many influencing factors involved, there is still a lack of comprehensive research on emergency intelligence capability evaluation system. In order to improve the rescue efficiency of major public health events, it is urgent to carry out in-depth research on the evaluation index system of emergency intelligence capability.

## 2. Related Works

### 2.1. Public Health Emergency Management Information

With the occurrence of emergencies in the real society, a variety of imperceptible risks appear. If the emergency is handled improperly, it will cause casualties, economic losses, ecological environment damage, and other serious consequences. In order to construct a scientific and perfect public health emergency management system, it is necessary to combine the matching intelligence support system. In recent years, more and more scholars have integrated emergency management and intelligence science to study emergency management intelligence, mainly involving three aspects: emergency management intelligence system, emergency intelligence decision optimization, and emergency intelligence cases. As for the emergency management intelligence system, Guo et al. summarized the features of the city emergency management information system as well as the difference with emergency decision-making information system through literature collection and case comparative analysis of the construction of urban emergency management intelligence activity model under the background of social modernity [1]; Jiang and Zhu discussed think tanks emergency intelligence service from the government's big data capacity model and proposed six constraints that affect the adjustment of four capability dimensions, at the same time to form a government big data capacity and then to adapt the think tanks emergency intelligence services [2]; Su and Jiang expounded the role of the information flow in each stage of the emergency response, which has to analyze the accurate description of the information flow in the three emergency stages of the epidemic prevention and then to reveal the overall evolution of the epidemic situation [3]. For decision-making optimization of emergency intelligence, Chen and Jiang designed emergency feature dictionary, emergency scenario database and strategy database, scenario map, strategy evaluation model, multiobjective optimization model to improve the research methods of intelligence collection, organization, processing, analysis, evaluation, and decision-making, thus providing intelligence support for emergency decision-making generation and optimization [4]; Li et al. proposed that the construction of the next generation of emergency intelligence was imminent, put forward some relevant path thinking from the perspective of “big intelligence” system, and made a deep thinking on the “restarting” of emergency intelligence from six aspects: resource, technology, personnel, coordination, decision-making, and science popularization [5]. In the case of emergency intelligence, Tang et al. conducted combining the function of emergency rapid response intelligence system by applying the case analysis method, introduced the architecture and main function of emergency rapid response intelligence system, and made a case study for emergency from warning linkage, network public opinion controlling, risk assessment, crisis identification, and warning by applying the intelligence system [6]; Liu and Su analyzed two types of natural disaster emergencies, namely Wenchuan earthquake and flood disaster in 2016. Through the review of the case content and with the help of emergency response information system, the two events are deeply analyzed in three phases. Decision-making suggestions for similar emergencies are proposed after the analysis [7]; Shen et al. analyzed toxic milk powder and blue-green algae from Taihu Lake to take public health events as the starting point, and the typical emergencies were analyzed in detail so as to provide relevant information and knowledge for dealing with emergencies [8].

### 2.2. Emergency Intelligence Capability Evaluation System

At present, China's emergency management and intelligence resources present a state of separation, and the role of emergency intelligence system to deal with major public health events has not been fully demonstrated. There are still many deficiencies in the overall construction of emergency intelligence capability evaluation system. The research on the evaluation of emergency intelligence capability mainly focuses on two aspects: the construction of the evaluation index system of emergency intelligence capability and the evaluation model of emergency intelligence capability, including Pan constructed security-related intelligence, emergency intelligence, emergency management, IT capability management, IS service quality evaluation, and their influencing factors, and established a model of EIS service capability and its influencing factors [9]; Chen analyzed the construction of emergency system from the perspective of colleges and universities, with the incubation period, outbreak period, spread period, and recovery period as the starting point and put forward the strategy of emergency system construction [10]; Han et al. constructed the overall theoretical framework of emergency intelligence capabilities for major public emergencies based on the perspective of intelligence process, dismantled and analyzed the components of think tank's emergency intelligence service capabilities, and put forward the service modes and service paths of think tank emergency intelligence service oriented to the difference of service object [11]; Guo and Zhang took COVID-19 as the specific problem, deduced the intelligence wisdom tree model of disease control emergency work, and constructed the corresponding evaluation system of intelligence ability [12]; Li and Sun summed up the evolution logic of the localization paradigm of the development of Chinese intelligence studies and intelligence work, from exclusive intelligence to the lack of intelligence and the “physical ability” of intelligence, as well as the development of Chinese intelligence studies and intelligence work with a deep branding of the times [13–15]. At present, there are relatively few studies on the analysis of emergency intelligence capability. Because of the difficulty in designing the evaluation index system, it is extremely important to construct a comprehensive, systematic, and standardized evaluation system of emergency intelligence capability for major public health events.

### 2.3. Evaluation Method of Emergency Intelligence Capability

The research of emergency intelligence capability evaluation focuses on the methods of emergency intelligence capability evaluation, mainly using mathematical evaluation method and statistical evaluation method. Mathematical evaluation methods include principal component analysis method, regression analysis method, data envelopment method, analytic hierarchy process, neural network method, gray system evaluation method, etc. Statistical analysis evaluation methods include descriptive statistical analysis evaluation method and inferential statistical analysis evaluation method. In terms of the implementation of evaluation methods, emergency intelligence capability involves a large number of practical problems combining subjective and objective, and most scholars use expert investigation method and in-depth interview method and expert scoring method to comprehensively evaluate the specific emergency intelligence capability. In recent years, decision-making methods based on uncertain language information have been widely studied and some achievements have been achieved. Some other methods have also been put forward to solve the problem of emergency intelligence. At present, the research on emergency intelligence is mainly analyzed from multiple perspectives, including collaborative perspective, national security perspective, and multiple research perspective. The use of research methods is less, including systems-theoretic accident modeling and process and block chain sharing, based on complex network and other methods.

Due to the inflexibility of questionnaire survey and expert interview design, the range of experts' answers is set in advance, and richer and more complete evaluation information cannot be obtained in the actual evaluation process. And the bias of expert evaluation cannot be reflected. Therefore, the evaluation of emergency intelligence capability of major public health events is not scientific and comprehensive. With the complexity of emergency intelligence of major public health events, relevant decision-makers need to make decisions within a limited time, and the evaluation information of emergency intelligence capacity of major public health events usually includes different sets of language terms. In order to meet the needs of actual decision-making situation, the evaluation information is represented by language value and corresponding probability, and the probabilistic uncertain language term set multiattribute decision-making method is used to evaluate the emergency intelligence capability of major public health events.

## 3. The Operational Mechanism of Emergency Intelligence Capability System for Major Public Health Events

### 3.1. The Connotation and Nature of Emergency Intelligence Capability of Major Public Health Events

Intelligence capability should be the comprehensive capability of information collection, information retrieval and storage, information analysis and research, information exchange and service, etc. It is a special set of application ability, with a certain level of characteristics. Emergency intelligence capability refers to the comprehensive quality of strategic information work by collecting, serving, processing, and guaranteeing information under certain environmental conditions after an emergency occurs. It is an important basic capability in the process of emergency management in China.

Compared with other intelligence, emergency intelligence of major public health events emphasizes the transformation of intelligence information, which transforms general information into useful information by analyzing original data. As the intelligence sources of major public health events are very extensive and diversified, emergency intelligence needs to integrate intelligence information from multiple sources, investigate the intelligence information, and judge whether major public health events occur based on data analysis. Therefore, the evaluation of emergency intelligence capability of major public health events requires the combination of objective data and subjective cognition. Objective data provide scientific interpretation and prediction of risks, while subjective cognition is used to process decision-makers' personal evaluation information.

### 3.2. Process of Defining Emergency Intelligence Capacity for Major Public Health Events

The construction of emergency intelligence system of major public health events needs to follow the evolution process of major public health events, including preparation period, response period, and recovery period. According to different stages, the definition of emergency intelligence capability corresponds to the content, and form and acquisition method of emergency intelligence has obvious differences. The process of defining intelligence capabilities for major public health events is shown in Figure 1.

#### 3.2.1. Emergency Intelligence Preparation Period

Emergency intelligence preparation period refers to when major public health events are in latent state. The epidemic has not yet broken out, and intelligence information has initially shown a crisis, but the epidemic has not spread widely, causing little damage, and the risk of the epidemic is not obvious. At this stage, the risk is not easily detected, the intelligence is difficult to obtain, the collection of emergency intelligence is not strong in purpose and pertinence, the demand for intelligence is wide, and the intelligence is difficult to collect. The main body of emergency intelligence collection in the preparatory period is the government public health department, which collects and analyzes information on various factors that may cause the epidemic through the initial emerging risks, and evaluates the risk of the epidemic [16].

#### 3.2.2. Emergency Intelligence Response Period

After the outbreak of major public health events, the epidemic keeps spreading, and the extent and scope of damage caused by major public health events keep expanding, which has a negative impact on people's physical and mental health and social stability and development. At this stage, the emergency ability of the intelligence system faces a severe test. The intelligence service personnel collect and collate the information related to the outbreak of major public health events in the shortest time and share information with medical institutions. During the response period of emergency intelligence, a large amount of epidemic-related intelligence collected during the preparation period of emergency intelligence should be screened and analyzed, and the quantity and quality of emergency intelligence should be emphasized to provide support for vaccine development and effectively control the development of the epidemic situation.

#### 3.2.3. Emergency Intelligence Recovery Period

The recovery period of emergency intelligence refers to that after the major public health events are controlled, the patients are treated effectively, the society is relatively stable, and the emergency intelligence is also relatively stable. In this stage, the quantity of emergency intelligence gradually decreases, and the intelligence collection in the recovery stage of emergency intelligence is more complete than the previous two stages. However, intelligence during the recovery period of emergency response intelligence is also important. It is necessary to trace the source of major public health events, analyze the losses caused by each stage of the epidemic, and summarize the experience and lessons brought by major public health events. At the same time, the recovery period of emergency intelligence should also collect information to prevent the recurrence of the epidemic, exchange emergency intelligence with international health organizations and governments, carry out global epidemic prevention, and maintain the stability of the recovery period.

### 3.3. The Operational Mechanism of Emergency Intelligence Capability System

The system of emergency intelligence capability is a chain structure with complexity and dynamics. According to the nature of major public health events, emergency management bodies in different professional fields are connected, including public health service, medical institutions, epidemic management centers, information service institutions, and World Health Organization. The emergency intelligence system identifies the collected emergency intelligence sources and obtains intelligence in the form of data, images, videos, texts, and audio through modern information technology and biometric technology, providing real-time epidemic information for emergency decision-making departments. Through the screening and analysis of emergency intelligence, the correctness and authority of emergency intelligence source channels are verified quickly and efficiently, and multisource intelligence is crosschecked through the combination of various intelligence processing technologies to ensure the rationality and accuracy of emergency intelligence required. After several rounds of screening of emergency intelligence, the emergency intelligence is compared with the previous case database, knowledge base, emergency model, and emergency strategy, and the emergency intelligence is integrated. Emergency intelligence is summarized into the corresponding classification database storage platform according to the characteristics of the type of emergency, development stage, and so on. In order to ensure that the required emergency intelligence is reasonable and accurate, the emergency management center will transfer the emergency intelligence to the specific service objects in a fast and appropriate way, directly and quickly play a role in emergency decision-making, continue to track major public health events, and adjust the emergency plan in time.

Under the background of digitization of social governance, the operation efficiency of emergency intelligence capability system determines the rescue efficiency of emergency management. The operation mechanism of the whole emergency intelligence capability highlights the systematic operation of the evolution of emergency intelligence system in each stage. Through the screening and aggregation of emergency intelligence, coordination and integration of multiparty emergency intelligence data resources, emergency decision-making tools, and emergency expert wisdom, the main body of emergency decision-making can quickly carry out rescue work of major public health events. It is beneficial to improve the efficiency of emergency management and plays a regulatory and promoting role in emergency management. The operation mechanism of the specific major public health emergency intelligence capability system is shown in Figure 2.

## 4. The Evaluation Index System for Emergency Intelligence Capability of Major Public Health Events

On the premise of ensuring the simplicity, comparability, flexibility, and comprehensiveness of the evaluation index system, a major public health emergency intelligence capability index system is designed to provide important decision-making support for government decision-making departments. In this paper, the structure of emergency intelligence capability of major public health events is divided into four dimensions, namely, emergency intelligence gathering capability, emergency intelligence processing capability, emergency intelligence service capability, and emergency intelligence guarantee capability. The specific major public health event emergency intelligence capability evaluation index system is shown in Table 1.

### 4.1. Emergency Intelligence Gathering Capability

Emergency intelligence collection capability refers to the comprehensive capability of collecting and acquiring intelligence information resources in major public health events through various information channels, providing emergency preparedness for subsequent emergency management and playing an early warning role. In the era of big data, public health departments, medical institutions, local think tanks, and social media can make use of modern information technology to obtain real-time information of major public health events, ensure the real-time and fast acquisition of emergency intelligence, and provide emergency intelligence support for emergency decision-making. The core elements of the ability of emergency intelligence collection include the completeness of emergency intelligence infrastructure, the sufficiency of basic workers of emergency intelligence, the ability of emergency intelligence support, and the ability of emergency intelligence supply.

### 4.2. Emergency Intelligence Service Capability

The ability of emergency intelligence service refers to the ability required by the decision-making body of emergency intelligence service during the whole process of emergency management from the outbreak to the end of major public health events. According to the specific content of emergency intelligence work at each stage of epidemic situation, the value of emergency intelligence service is integrated into the integration and coordination of information work in the whole process of emergency management. It includes the ability of participating in emergency intelligence information, supporting emergency intelligence, sharing emergency intelligence, and developing emergency intelligence continuously.

### 4.3. Emergency Intelligence Processing Capability

The ability of emergency intelligence processing refers to the ability of analyzing and processing emergency intelligence. Each decision-making department carries the intelligence transfer, the analysis, the communication, the exchange to the intelligence, the screening, and the collation to the emergency intelligence. After identifying the accuracy of emergency intelligence of major public health events, the response level of major public health events is determined. It involves the ease of use, security, and responsiveness of emergency intelligence. In the process of intelligence processing, information communication and cooperation between various intelligence departments are emphasized, and whether the emergency intelligence is submitted quickly and accurately, the intelligence is released in time and through various channels is emphasized.

### 4.4. Emergency Intelligence Guarantee Capability

Emergency intelligence support capability refers to the ability to maintain orderly information activities of emergency departments and ensure the smooth development of emergency rescue work after the occurrence of major public health events. This stage mainly includes emergency intelligence policy support capability, emergency intelligence funding support capability, and emergency intelligence technology support capability.

## 5. Proposed Model

### 5.1. Some Concepts Related to PULTS

In order to express the preference of experts more accurately and deal with the intelligence in the emergency decision-making process of major public health events effectively, it is necessary to deal with the demand of actual decision-making situation. In this paper, probabilistic uncertain language term set (PULTS) with VIKOR multiattribute decision-making method is used to evaluate the emergency intelligence capability of major public health events. VIKOR is a multiattribute evaluation method for complex systems, which is characterized by maximizing “group utility” and minimizing “individual regret.”

**Definition 1 .**

[17] Let *S*={*S*_*t*_*|t*=−*τ*,…, −1,0,1,…, *τ*} be a language term set, then the PULTS can be expressed as:

(1) $$\begin{array}{c} S\left(p\right)=\left\{\langle \left[s_{L^{\lambda }}^{\lambda },s_{U^{\lambda }}^{\lambda }\right],p^{\lambda }\rangle |p\geq 0,\lambda =1,2,\ldots ,l,\sum_{\lambda =1}^{l}p^{\lambda }\leq 1\right\}, \end{array}$$

where [*s*_*L*_^*λ*^, *s*_*U*_^*λ*^] is the *λ* th uncertain language set in *S*(*p*) and satisfies *s*_*L*_^*λ*^ < *s*_*U*_^*λ*^, probability *p*^*λ*^ is the possibility of occurrence of [*s*_*L*_^*λ*^, *s*_*U*_^*λ*^], and *l* is the number of elements in *S*(*p*).

**Definition 2 .**

[17] Let *P*_1_={*a*_*i*_*|i*=0,1,…, #*P*_1_}, *a*_*i*_=*s*_[*a*_*i*_^−^, *a*_*i*_^+^]_(*p*_*i*_) and *P*_2_={*b*_*j*_*|j*=0,1,…, #*P*_2_}, *b*_*j*_=*s*_[*b*_*j*_^−^, *b*_*j*_^+^]_(*p*_*j*_) be two arbitrary PULTSs and #*P*_1_=#*P*_2_, then the distance can be calculated by:

(2) $$\begin{array}{c} d\left(P_{1},P_{2}\right)=\frac{1}{2\tau }\left(\sqrt{\frac{\sum_{i=0}^{\#P_{1}}{\left(p_{i}a_{i}^{-}-q_{j}b_{j}^{-}\right)}^{2}}{\#P_{1}}}+\sqrt{\frac{\sum_{i=0}^{\#P_{1}}{\left(p_{i}a_{i}^{+}-q_{j}b_{j}^{+}\right)}^{2}}{\#P_{1}}}\right). \end{array}$$

**Definition 3 .**

[17] Let *P*_1_={*a*_*i*_*|i*=0,1,…, #*P*_1_}, *a*_*i*_=*s*_[*a*_*i*_^−^, *a*_*i*_^+^]_(*p*_*i*_) be a PULTS, then the score value function and deviation degree function are defined as:

(3) $$\begin{array}{c} E\left(P\right)=\frac{\sum_{i=0}^{\#P}\left(a_{i}^{+}+a_{i}^{-}\right)p_{i}}{2\sum_{i=0}^{\#P}p_{i}},a\\ V\left(P\right)=\frac{1}{\sum_{i=0}^{\#P}p_{i}}\left(\frac{1}{2}\sqrt{\sum_{i=0}^{\#P}p_{i}\left(a_{i}^{+}-a_{i}^{-}\right)}+\sqrt{\sum_{i=0}^{\#P}p_{i}{\left(\frac{a_{i}^{+}+a_{i}^{-}}{2}-E\left(p\right)\right)}^{2}}\right). \end{array}$$

Two PULTSs can be compared according to the score function and deviation degree function. Given any two PULTS *P*_1_ and *P*_2_, the following comparative conclusions can be drawn:

1. If *E*(*P*_1_) < *E*(*P*_2_), then *P*_1_ < *P*_2_.
2. If *E*(*P*_1_) > *E*(*P*_2_), then *P*_1_ > *P*_2_.
3. If *E*(*P*_1_)=*E*(*P*_2_), then *P*_1_=*P*_2_.
4. If *V*(*P*_1_) < *V*(*P*_2_), then *P*_1_ < *P*_2_.
5. If *V*(*P*_1_) > *V*(*P*_2_), then *P*_1_ > *P*_2_.
6. If *V*(*P*_1_)=*V*(*P*_2_), then *P*_1_=*P*_2_.

### 5.2. Problem Description

Assuming that a major public health event occurs in a certain region, the emergency intelligence capability of major public health event is now evaluated. There is a candidate city *X*={*x*_1_, *x*_2_,…, *x*_*m*_} for emergency intelligence capability evaluation in this region, which has *n* evaluation indexes *C*={*C*_1_, *C*_2_,…, *C*_*n*_} with known attribute weights *w*={*w*_1_, *w*_2_,…, *w*_*n*_} and ∑_*i*=1_^*n*^*w*_*i*_=1,  0 ≤ *w*_*i*_ ≤ 1. The language term set corresponding to expert evaluation information is *S*={*s*_*i*_*|i*=0,1,2,…, 2*τ*}. Following the principle of maximization of group utility and minimization of individual regret, experts scored each index of candidate cities for evaluation of emergency intelligence capability of major public health events and then obtained the probabilistic uncertain language matrix *F*=(*f*_*ij*_)_*m*×*n*_, where *f*_*ij*_ represents the expert's evaluation of each candidate city *x*_*i*_(*i*=1,2,…, *m*) for emergency response intelligence capability evaluation under each evaluation index *C*_*j*_(*j*=1,2,…, *n*).

### 5.3. VIKOR

VIKOR method is a compromise decision-making method proposed by Opricovic (1998) based on the limitations of TOPSIS method. Its core idea is to determine the compromise optimal solution which is closest to the positive ideal solution and farthest from the negative ideal solution through computational analysis. By defining maximization of group utility and minimization of individual regret, ranking the advantages and disadvantages of a limited number of candidate schemes can be applied to multiattribute decision-making problems in which decision-makers cannot or do not know how to express preferences accurately, there may be conflicts among evaluation attributes, and decision-makers can accept compromise schemes. The basic process is as follows: (1) build the initial decision matrix; (2) identify positive and negative ideal solutions; (3) determine the maximum group utility value and the maximum individual regret value; (4) calculate trade-off value.

### 5.4. The Decision-Making Procedure

We use the VIKOR multiattribute decision-making method to solve the problem of emergency intelligence capability evaluation of major public health events in probabilistic uncertain language environment. Experts gave the evaluation value *f*_*ij*_ and obtained an initial decision matrix of *m* × *n*, which is denoted as *F*=(*f*_*ij*_)_*m*×*n*_:

(4) $$\begin{array}{c} F={\left(f_{ij}\right)}_{m\times n}=\left[\begin{array}{cccc} P\left(x_{1}|C_{1}\right) & P\left(x_{1}|C_{2}\right) & \ldots & P\left(x_{1}|C_{n}\right)\\ P\left(x_{2}|C_{1}\right) & P\left(x_{2}|C_{2}\right) & \ldots & P\left(x_{2}|C_{n}\right)\\ \ldots & \ldots & \ldots & \ldots \\ P\left(x_{m}|C_{1}\right) & P\left(x_{m}|C_{2}\right) & \ldots & P\left(x_{m}|C_{n}\right) \end{array}\right]. \end{array}$$

The main operation steps are as follows:

Step 1: Calculate the score value matrix and the deviation degree matrix. According to equations (3) and (4), score value matrix and deviation degree matrix are calculated.
Step 2: Determine positive and negative ideal solutions. The optimal value and the worst value of each attribute are determined for the candidate cities of emergency intelligence capability evaluation. Under the benefit attribute, the positive and negative ideal solutions are:
  (5) $$\begin{array}{c} f_{j}^{+}=\underset{i}{\max}\left\{f_{ij},\;i=1,2,\ldots ,m\right\},\\ f_{j}^{-}=\underset{i}{\min}\left\{f_{ij},\;i=1,2,\ldots ,m\right\}. \end{array}$$
Under the cost attribute, the positive and negative ideal solutions are:
  (6) $$\begin{array}{c} f_{j}^{+}=\underset{i}{\min}\left\{f_{ij},\;i=1,2,\ldots ,m\right\},\\ f_{j}^{-}=\underset{i}{\max}\left\{f_{ij},\;i=1,2,\ldots ,m\right\}. \end{array}$$
The relatively positive ideal solution and relatively negative ideal solution can be obtained as follows:
  (7) $$\begin{array}{c} X^{+}≜\left(f_{1}^{+},f_{2}^{+},\ldots ,f_{n}^{+}\right),\\ X^{-}≜\left(f_{1}^{-},f_{2}^{-},\ldots ,f_{n}^{-}\right). \end{array}$$
Step 3: Determine group utility *S*_*i*_ and maximum individual regret *R*_*i*_ among *n* attributes of each candidate city for emergency intelligence capability evaluation:
  (8) $$\begin{array}{c} S_{i}=\sum_{j=1}^{n}\frac{w_{j}\left(Ef_{j}^{+}-Ef_{ij}\right)}{Ef_{j}^{+}-Ef_{ij}},\;i=1,2,\ldots ,m,\\ R_{i}=\max\left[\frac{w_{j}\left(Ef_{j}^{+}-Ef_{ij}\right)}{Ef_{j}^{+}-Ef_{ij}},\;j=1,2,\ldots ,n\right],\;i=1,2,\ldots ,m. \end{array}$$
Step 4: Calculate the value of the compromise function *Q*_*i*_:
  (9) $$\begin{array}{c} Q_{j}=\frac{v\left(S_{j}-S^{*}\right)}{S^{-}-S^{*}}+\frac{\left(1-v\right)\left(R_{j}-R^{*}\right)}{R^{-}-R^{*}}. \end{array}$$
where *S*^*∗*^=min_1≤*j*≤*m*_*S*_*j*_, *S*^−^=max_1≤*j*≤*m*_*S*_*j*_, *R*^*∗*^=min_1≤*j*≤*m*_*R*_*j*_, *R*^−^=max_1≤*j*≤*m*_*R*_*j*_ and *v* is expressed as a decision-making mechanism coefficient, if *v* > 0.5, then said according to maximize the effects of group decision-making mechanism. If *v* < 0.5, then minimize the decision-making mechanism of individual regret values; if *v*=0.5, then according to the largest group negotiated effect and minimum individual regret value are equally important decision-making mechanism to make decisions.
Step 5: Sort. On the basis of *S*_*i*_, *R*_*i*_, and *Q*_*i*_, the optimal solution can be obtained by sorting according to VIKOR's criteria.

In this section, the VIKOR method for PULTSs model for evaluation criteria for emergency intelligence capacity will be built, as shown in Figure 3.

## 6. Case Study

Because of the complexity of the problem itself or the limitation of the expert's cognitive level, decision information inevitably contains uncertainty. Traditional methods require decision-makers to express information as a certain predefined language term. It is difficult to achieve in a complex and uncertain environment. Uncertain language expressions contain multiple terms directly or indirectly, and each term may be the truth value of language variables, which is more consistent with the language habit of expressing uncertainty.

The current COVID-19 outbreak poses a huge challenge to global health governance. It is of great significance to establish and perfect emergency intelligence management system to evaluate emergency intelligence capability scientifically and reasonably. In order to illustrate the feasibility and effectiveness of the method, this section takes COVID-19 epidemic as the background and selects four cities *X*_*i*_(*i*=1,2,3,4) as examples to evaluate the emergency intelligence capability under the COVID-19 epidemic. The evaluation team is composed of experts from local public health departments, medical institutions, epidemic management centers, and information service institutions. And the expert members of the evaluation team are invited to score the indicators of emergency response intelligence capability of each city based on their own professional knowledge. In order to express the evaluation information more directly and comprehensively, we propose a 9-value scale in probabilistic uncertain language environment, as *S*={*s*_0_, *s*_1_, *s*_2_, *s*_3_, *s*_4_, *s*_5_, *s*_6_, *s*_7_, *s*_8_}. Through unified collection and processing, the initial matrix is normalized and the normalized matrix is obtained, as shown in Table 2.

The specific evaluation steps are as follows:

  Step 1: Calculate the score value matrix and the deviation degree matrix. By using equations (3) and (4), score value matrix and deviation degree matrix are obtained, as shown in Tables 3 and 4.
  Step 2: Calculate the positive and negative ideal solutions. According to the score value matrix and the deviation degree matrix, positive ideal solution and negative ideal solution of indicators at all levels can be obtained, as shown in Tables 5 and 6.
  Step 3: Calculate maximum group utility value and maximum individual regret value. Equations (5) and (6) are used to determine the group utility and the maximum individual regret among the attributes of each candidate scheme, as shown in Table 7. The minimum value of the maximum group utility value is *X*_1_, and the minimum value of the maximum individual regret value is *X*_2_. Therefore, according to the judgment criteria of VIKOR method, there is no stable optimal candidate city in these four cities, and there is a compromise solution set.
  Step 4: Calculate the value of the compromise function. In order to facilitate comprehensive comparative analysis, formula (7) is used to calculate the compromise values under each decision coefficient, as shown in Table 8.
  Step 5: Sort. According to the judgment criteria of VIKOR method, the sorting results are obtained as shown in Table 9.

According to Table 9, in the case of compromise solutions, different decision coefficients will lead to different decision results. In the mechanism of strengthening individual regret, *X*_2_ was slightly better than *X*_1_, and the comprehensive ranking result was *X*_2_≻*X*_1_≻*X*_3_≻*X*_4_. Under the compromise equilibrium mechanism, the comprehensive ranking result is *X*_2_≻*X*_1_≻*X*_4_≻*X*_3_; that is, the city with the optimal emergency intelligence capability is *X*_2_. The comprehensive ranking result obtained under the enhanced group utility mechanism is *X*_2_≻*X*_1_≻*X*_4_≻*X*_3_, *X*_2_ is slightly better than *X*_1_, and at this time, the city with the optimal emergency intelligence capability is *X*_2_. In general, the emergency intelligence capability of *X*_1_ and *X*_2_ is better than *X*_3_ and *X*_4_, which provides evaluation criteria for the emergency intelligence capability of *X*_3_ and *X*_4_ for major public health events in the future and strengthens the construction and improvement of each emergency intelligence capability, so as to carry out emergency rescue work more quickly and effectively.

## 7. Conclusion

Based on the construction of the evaluation system of emergency intelligence capability for major public health events, we make a scientific evaluation of the system of emergency intelligence capability full of uncertainty and complexity, considering the cognitive limitations and fuzzy thinking of decision-makers. To achieve the unity of emergency intelligence and scientific decision-making, building VIKOR based on multiple attribute decision-making method is a major public health event emergency intelligence capability multiattribute evaluation model. At present, the research on probabilistic linguistic fuzzy set theory is still in the exploratory stage. Although some scholars have made some achievements, there are still many aspects worthy of study, and there are some deficiencies in the existing research. The quantitative index is introduced into the construction of real estate investment decision-making index system, and each index is considered. The correlation between criteria is integrated into the decision model. In the future, quantitative indicators will be introduced into the construction of the evaluation index system of emergency intelligence capability, and the correlation between indicators will be incorporated into the decision-making model.

## Figures and Tables

**Figure 1:** Process definition diagram of emergency intelligence capability for major public health events.

**Figure 2:** The operational mechanism of emergency intelligence capability system for major public health events.

**Figure 3:** The flowchart of the VIKOR method for PULTSs model.

**Table 1:** Evaluation index system of emergency intelligence capability of major public health events.

		First-level indicators	Second-level indicators
Evaluation of emergency intelligence capability of major public health events
		Emergency intelligence gathering capability (*C*_1_)	The completeness of emergency intelligence infrastructure (*C*_11_)
			The sufficiency of basic workers for emergency intelligence (*C*_12_)
			Emergency intelligence support capability (*C*_13_)
			Emergency intelligence supply capability(*C*_14_)
		Emergency intelligence service capability (*C*_2_)	Emergency intelligence participation capability (*C*_21_)
			Emergency intelligence support capability (*C*_22_)
			Emergency intelligence coordination and sharing capability (*C*_23_)
			Emergency intelligence continuous development capability (*C*_24_)
		Emergency intelligence processing capability (*C*_3_)	Information transmission capability of emergency intelligence (*C*_31_)
			Information analysis capability of emergency intelligence (*C*_32_)
			Information processing capability of emergency intelligence (*C*_33_)
			Information analysis efficiency of emergency intelligence (C_34_)
			Ease of use of emergency intelligence information (C_35_)
			Security of emergency intelligence information (*C*_36_)
			Responsiveness of emergency intelligence information (*C*_37_)
			Information reporting capability of emergency intelligence (*C*_38_)
			Timeliness of reporting emergency intelligence (*C*_39_)
			Intelligence communication between emergency services (*C*_310_)
			Intelligence collaboration between emergency services (*C*_311_)
			Diversity of emergency intelligence release channels (*C*_312_)
		Emergency intelligence support capability (*C*_4_)	Emergency intelligence policy support capability (*C*_41_)
			Emergency intelligence financial support capability (*C*_42_)
			Emergency intelligence technology support capability (*C*_43_)

**Table 2:** Normalized evaluation matrix.

	*X*_1_	*X*_2_	*X*_3_	*X*_4_
*C*_11_	{[*S*_3_, *S*_4_](0.4), [*S*_4_, *S*_5_](0.4), [*S*_5_, *S*_5_](0.2)}	{[*S*_3_, *S*_4_](0.5), [*S*_4_, *S*_5_](0.5), [*S*_3_, *S*_4_](0.0)}	{[*S*_3_, *S*_4_](0.4), [*S*_4_, *S*_5_](0.4), [*S*_5_, *S*_5_](0.2)}	{[*S*_3_, *S*_4_](0.4), [*S*_4_, *S*_5_](0.4), [*S*_5_, *S*_5_](0.2)}
*C*_12_	{[*S*_3_, *S*_4_](0.4), [*S*_4_, *S*_4_](0.6), [*S*_3_, *S*_4_](0.0)}	{[*S*_4_, *S*_5_](0.4), [*S*_4_, *S*_6_](0.4), [*S*_5_, *S*_5_](0.2)}	{[*S*_4_, *S*_6_](0.5), [*S*_5_, *S*_6_](0.5), [*S*_4_, *S*_6_](0.0)}	{[*S*_4_, *S*_5_](0.2), [*S*_4_, *S*_6_](0.6), [*S*_5_, *S*_6_](0.2)}
*C*_13_	{[*S*_4_, *S*_6_](0.3), [*S*_5_, *S*_7_](0.7), [*S*_4_, *S*_6_](0.0)}	{[*S*_5_, *S*_5_](0.2), [*S*_5_, *S*_6_](0.5), [*S*_5_, *S*_7_](0.3)}	{[*S*_5_, *S*_5_](0.3), [*S*_5_, *S*_6_](0.4), [*S*_5_, *S*_7_](0.3)}	{[*S*_5_, *S*_5_](0.5), [*S*_5_, *S*_6_](0.5), [*S*_5_, *S*_5_](0.0)}
*C*_14_	{[*S*_5_, *S*_7_](0.1), [*S*_6_, *S*_6_](0.4), [*S*_6_, *S*_7_](0.5)}	{[*S*_5_, *S*_6_](0.3), [*S*_6_, *S*_7_](0.7), [*S*_5_, *S*_6_](0.0)}	{[*S*_5_, *S*_6_](1.0), [*S*_5_, *S*_6_](0.0), [*S*_5_, *S*_6_](0.0)}	{[*S*_5_, *S*_7_](0.2), [*S*_6_, *S*_6_](0.3), [*S*_6_, *S*_7_](0.5)}
*C*_21_	{[*S*_5_, *S*_6_](0.2), [*S*_5_, *S*_7_](0.6), [*S*_6_, *S*_6_](0.2)}	{[*S*_6_, *S*_6_](0.2), [*S*_6_, *S*_7_](0.6), [*S*_7_, *S*_7_](0.2)}	{[*S*_5_, *S*_6_](0.3), [*S*_5_, *S*_7_](0.7), [*S*_5_, *S*_6_](0.0)}	{[*S*_5_, *S*_7_](0.4), [*S*_5_, *S*_6_](0.4), [*S*_6_, *S*_6_](0.2)}
*C*_22_	{[*S*_6_, *S*_7_](0.7), [*S*_7_, *S*_7_](0.3)[*S*_6_, *S*_7_](0.0)}	{[*S*_6_, *S*_6_](1.0), [*S*_6_, *S*_6_](0.0), [*S*_6_, *S*_6_](0.0)}	{[*S*_5_, *S*_5_](0.6), [*S*_5_, *S*_6_](0.4), [*S*_5_, *S*_5_](0.0)}	{[*S*_4_, *S*_6_](0.5), [*S*_6_, *S*_6_](0.2), [*S*_5_, *S*_6_](0.3)}
*C*_23_	{[*S*_6_, *S*_6_](0.2), [*S*_6_, *S*_7_](0.8), [*S*_6_, *S*_6_](0.0)}	{[*S*_5_, *S*_5_](0.2), [*S*_5_, *S*_6_](0.3), [*S*_5_, *S*_7_](0.5)}	{[*S*_5_, *S*_5_](0.4), [*S*_5_, *S*_6_](0.2), [*S*_5_, *S*_7_](0.4)}	{[*S*_5_, *S*_5_](0.4), [*S*_5_, *S*_6_](0.4), [*S*_5_, *S*_7_](0.2)}
*C*_24_	{[*S*_5_, *S*_6_](1.0), [*S*_5_, *S*_6_](0.0), [*S*_5_, *S*_6_](0.0)}	{[*S*_5_, *S*_7_](0.4), [*S*_6_, *S*_6_](0.4), [*S*_5_, *S*_7_](0.2)}	{[*S*_4_, *S*_5_](0.4), [*S*_4_, *S*_6_](0.3), [*S*_4_, *S*_7_](0.3)}	{[*S*_5_, *S*_6_](0.6), [*S*_6_, *S*_6_](0.3), [*S*_6_, *S*_7_](0.1)}
*C*_31_	{[*S*_4_, *S*_5_](0.1), [*S*_5_, *S*_5_](0.4), [*S*_5_, *S*_6_](0.5)}	{[*S*_4_, *S*_5_](0.4), [*S*_4_, *S*_6_](0.6), [*S*_4_, *S*_5_](0.0)}	{[*S*_5_, *S*_5_](0.4), [*S*_5_, *S*_6_](0.4), [*S*_6_, *S*_6_](0.2)}	{[*S*_5_, *S*_5_](0.3), [*S*_5_, *S*_6_](0.5), [*S*_6_, *S*_6_](0.2)}
*C*_32_	{[*S*_4_, *S*_5_](0.8), [*S*_5_, *S*_5_](0.2), [*S*_4_, *S*_5_](0.0)}	{[*S*_4_, *S*_5_](0.4), [*S*_4_, *S*_6_](0.6), [*S*_4_, *S*_5_](0.0)}	{[*S*_5_, *S*_5_](0.5), [*S*_5_, *S*_6_](0.5), [*S*_5_, *S*_5_](0.0)}	{[*S*_5_, *S*_5_](0.4), [*S*_5_, *S*_6_](0.6), [*S*_5_, *S*_5_](0.0)}
*C*_33_	{[*S*_4_, *S*_5_](0.4), [*S*_5_, *S*_5_](0.4), [*S*_5_, *S*_6_](0.2)}	{[*S*_4_, *S*_5_](1.0), [*S*_4_, *S*_5_](0.0), [*S*_4_, *S*_5_](0.0)}	{[*S*_4_, *S*_5_](0.5), [*S*_5_, *S*_5_](0.2), [*S*_5_, *S*_6_](0.3)}	{[*S*_4_, *S*_5_](0.9), [*S*_5_, *S*_5_](0.1), [*S*_4_, *S*_5_](0.0)}
*C*_34_	{[*S*_4_, *S*_4_](0.2), [*S*_4_, *S*_5_](0.8), [*S*_4_, *S*_4_](0.0)}	{[*S*_4_, *S*_4_](0.2), [*S*_4_, *S*_5_](0.8), [*S*_4_, *S*_4_](0.0)}	{[*S*_4_, *S*_4_](0.3), [*S*_4_, *S*_5_](0.5), [*S*_5_, *S*_4_](0.2)}	{[*S*_4_, *S*_4_](0.4), [*S*_4_, *S*_5_](0.6), [*S*_4_, *S*_4_](0.0)}
*C*_35_	{[*S*_4_, *S*_6_](0.3), [*S*_5_, *S*_5_](0.7), [*S*_4_, *S*_5_](0.0)}	{[*S*_5_, *S*_6_](0.4), [*S*_5_, *S*_7_](0.6), [*S*_5_, *S*_6_](0.0)}	{[*S*_4_, *S*_6_](0.3), [*S*_4_, *S*_7_](0.5), [*S*_5_, *S*_6_](0.2)}	{[*S*_5_, *S*_6_](0.5), [*S*_5_, *S*_7_](0.5)[*S*_5_, *S*_6_](0.0)}
*C*_36_	{[*S*_4_, *S*_6_](0.4), [*S*_5_, *S*_5_](0.6), [*S*_4_, *S*_5_](0.0)}	{[*S*_5_, *S*_5_](0.5), [*S*_5_, *S*_6_](0.5), [*S*_5_, *S*_5_](0.0)}	{[*S*_4_, *S*_5_](0.2), [*S*_5_, *S*_5_](0.3), [*S*_5_, *S*_6_](0.5)}	{[*S*_4_, *S*_5_](0.6), [*S*_4_, *S*_5_](0.3), [*S*_5_, *S*_5_](0.1)}
*C*_37_	{[*S*_4_, *S*_5_](0.2), [*S*_5_, *S*_5_](0.4), [*S*_5_, *S*_6_](0.4)}	{[*S*_4_, *S*_5_](0.3), [*S*_5_, *S*_5_](0.4), [*S*_5_, *S*_6_](0.3)}	{[*S*_4_, *S*_5_](0.5), [*S*_5_, *S*_5_](0.5), [*S*_4_, *S*_5_](0.0)}	{[*S*_4_, *S*_5_](0.6), [*S*_5_, *S*_5_](0.4), [*S*_5_, *S*_6_](0.0)}
*C*_38_	{[*S*_4_, *S*_5_](0.3), [*S*_5_, *S*_5_](0.3), [*S*_5_, *S*_6_](0.4)}	{[*S*_4_, *S*_5_](0.2), [*S*_4_, *S*_6_](0.4), [*S*_5_, *S*_6_](0.4)}	{[*S*_4_, *S*_5_](0.2), [*S*_4_, *S*_6_](0.4), [*S*_5_, *S*_6_](0.4)}	{[*S*_4_, *S*_5_](0.1), [*S*_4_, *S*_6_](0.3), [*S*_5_, *S*_6_](0.6)}
*C*_39_	{[*S*_4_, *S*_5_](0.2), [*S*_5_, *S*_5_](0.4), [*S*_5_, *S*_6_](0.4)}	{[*S*_4_, *S*_6_](0.2), [*S*_5_, *S*_6_](0.8), [*S*_4_, *S*_6_](0.0)}	{[*S*_4_, *S*_6_](0.5), [*S*_5_, *S*_5_](0.3), [*S*_5_, *S*_6_](0.2)}	{[*S*_4_, *S*_6_](0.1), [*S*_5_, *S*_6_](0.9), [*S*_4_, *S*_6_](0.0)}
*C*_310_	{[*S*_4_, *S*_5_](0.2), [*S*_5_, *S*_6_](0.8), [*S*_4_, *S*_5_](0.0)}	{[*S*_4_, *S*_5_](0.3), [*S*_5_, *S*_5_](0.3), [*S*_5_, *S*_6_](0.4)}	{[*S*_4_, *S*_5_](0.3), [*S*_5_, *S*_5_](0.7), [*S*_4_, *S*_5_](0.0)}	{[*S*_4_, *S*_5_](0.2), [*S*_5_, *S*_5_](0.3), [*S*_5_, *S*_6_](0.5)}
*C*_311_	{[*S*_4_, *S*_6_](0.6), [*S*_5_, *S*_6_](0.4), [*S*_4_, *S*_6_](0.0)}	{[*S*_5_, *S*_6_](0.2), [*S*_6_, *S*_6_](0.4), [*S*_6_, *S*_7_](0.4)}	{[*S*_5_, *S*_6_](0.2), [*S*_6_, *S*_6_](0.5), [*S*_6_, *S*_7_](0.3)}	{[*S*_5_, *S*_6_](0.3), [*S*_6_, *S*_6_](0.5), [*S*_6_, *S*_7_](0.2)}
*C*_312_	{[*S*_4_, *S*_6_](0.2), [*S*_5_, *S*_5_](0.5), [*S*_5_, *S*_7_](0.3)}	{[*S*_4_, *S*_6_](0.5), [*S*_5_, *S*_6_](0.4), [*S*_4_, *S*_5_](0.1)}	{[*S*_4_, *S*_5_](0.3), [*S*_5_, *S*_5_](0.5), [*S*_5_, *S*_6_](0.2)}	{[*S*_4_, *S*_5_](0.3), [*S*_5_, *S*_5_](0.7), [*S*_4_, *S*_5_](0.0)}
*C*_41_	{[*S*_5_, *S*_6_](0.2), [*S*_6_, *S*_7_](0.8), [*S*_5_, *S*_6_](0.0)}	{[*S*_5_, *S*_5_](0.2), [*S*_5_, *S*_6_](0.6), [*S*_5_, *S*_7_](0.2)}	{[*S*_5_, *S*_5_](0.3), [*S*_5_, *S*_6_](0.5), [*S*_5_, *S*_7_](0.2)}	{[*S*_5_, *S*_5_](0.1), [*S*_5_, *S*_6_](0.4), [*S*_5_, *S*_7_](0.5)}
*C*_42_	{[*S*_5_, *S*_6_](1.0), [*S*_5_, *S*_6_](0.0), [*S*_5_, *S*_6_](0.0)}	{[*S*_5_, *S*_6_](0.3), [*S*_6_, *S*_6_](0.7), [*S*_5_, *S*_6_](0.0)}	{[*S*_5_, *S*_6_](0.5), [*S*_6_, *S*_6_](0.5), [*S*_5_, *S*_6_](0.0)}	{[*S*_5_, *S*_6_](0.3), [*S*_6_, *S*_6_](0.3), [*S*_6_, *S*_7_](0.4)}
*C*_43_	{[*S*_5_, *S*_6_](0.8), [*S*_6_, *S*_6_](0.2), [*S*_5_, *S*_6_](0.0)}	{[*S*_5_, *S*_6_](1.0), [*S*_5_, *S*_6_](0.0), [*S*_5_, *S*_6_](0.0)}	{[*S*_5_, *S*_5_](0.4), [*S*_5_, *S*_6_](0.3), [*S*_6_, *S*_6_](0.3)}	{[*S*_5_, *S*_7_](0.4), [*S*_6_, *S*_6_](0.6), [*S*_5_, *S*_6_](0.0)}

**Table 3:** The score value matrix of probabilistic uncertain languages.


$E\left[F\right]=\left[\begin{array}{cccc} 4.15 & 4.00 & 4.20 & 4.00\\ 4.20 & 5.25 & 5.55 & 4.95\\ 5.25 & 5.25 & 5.70 & 5.25\\ 6.25 & 6.20 & 5.55 & 6.25\\ 5.80 & 6.50 & 5.85 & 5.80\\ 6.25 & 6.00 & 5.20 & 5.45\\ 6.00 & 5.60 & 5.60 & 5.40\\ 5.50 & 6.15 & 4.95 & 5.70\\ 4.60 & 4.80 & 5.40 & 5.40\\ 4.90 & 5.00 & 5.20 & 5.30\\ 4.50 & 4.50 & 4.90 & 4.50\\ 5.00 & 4.40 & 4.45 & 4.30\\ 5.20 & 5.80 & 5.35 & 5.70\\ 5.10 & 5.25 & 4.75 & 4.80\\ 4.85 & 5.00 & 5.15 & 4.70\\ 5.20 & 5.10 & 4.85 & 5.25\\ 5.30 & 5.20 & 5.10 & 5.45\\ 6.20 & 5.25 & 5.15 & 5.15\\ 5.20 & 6.10 & 6.00 & 5.90\\ 5.30 & 4.75 & 4.95 & 4.85\\ 6.20 & 4.85 & 4.75 & 4.95\\ 5.60 & 5.75 & 5.85 & 5.50\\ 5.40 & 5.50 & 5.60 & 6.00 \end{array}\right]$

**Table 4:** The deviation degree matrix of probabilistic uncertain languages.


$V\left[F\right]=\left[\begin{array}{cccc} 1.05 & 1.00 & 0.81 & 0.80\\ 0.58 & 0.98 & 1.05 & 1.15\\ 1.25 & 1.20 & 1.06 & 0.55\\ 0.75 & 0.95 & 0.55 & 0.85\\ 1.06 & 0.73 & 1.85 & 1.02\\ 0.65 & 0.00 & 1.20 & 1.45\\ 0.65 & 1.15 & 0.60 & 0.75\\ 0.50 & 0.92 & 0.68 & 0.70\\ 0.72 & 1.08 & 0.82 & 0.68\\ 0.64 & 0.78 & 0.60 & 0.63\\ 0.50 & 0.50 & 1.12 & 0.62\\ 0.50 & 0.64 & 1.45 & 0.63\\ 0.72 & 1.08 & 0.69 & 1.04\\ 0.64 & 0.75 & 0.60 & 0.92\\ 0.76 & 0.50 & 0.88 & 0.64\\ 0.65 & 0.65 & 0.75 & 0.63\\ 0.85 & 1.20 & 1.20 & 1.02\\ 0.85 & 0.82 & 0.95 & 0.80\\ 0.90 & 0.76 & 0.73 & 0.70\\ 1.15 & 0.75 & 0.75 & 0.55\\ 0.90 & 0.85 & 0.80 & 1.15\\ 0.50 & 0.75 & 0.85 & 0.82\\ 0.48 & 0.50 & 0.68 & 0.62 \end{array}\right]$

**Table 5:** Positive ideal solutions for probabilistic uncertain languages.


$X^{+}=\left[\begin{array}{c} \left\{\left[S_{3},S_{4}\right]\left(0.4\right),\left[S_{4},S_{5}\right]\left(0.4\right),\left[S_{5},S_{5}\right]\left(0.2\right)\right\}\\ \left\{\left[S_{4},S_{6}\right]\left(0.5\right),\left[S_{5},S_{6}\right]\left(0.5\right),\left[S_{4},S_{6}\right]\left(0.0\right)\right\}\\ \left\{\left[S_{4},S_{6}\right]\left(0.3\right),\left[S_{5},S_{7}\right]\left(0.7\right),\left[S_{4},S_{6}\right]\left(0.0\right)\right\}\\ \left\{\left[S_{5},S_{7}\right]\left(0.2\right),\left[S_{6},S_{6}\right]\left(0.2\right),\left[S_{6},S_{7}\right]\left(0.6\right)\right\}\\ \left\{\left[S_{6},S_{6}\right]\left(0.2\right),\left[S_{6},S_{7}\right]\left(0.6\right),\left[S_{7},S_{7}\right]\left(0.2\right)\right\}\\ \left\{\left[S_{6},S_{7}\right]\left(0.7\right),\left[S_{7},S_{7}\right]\left(0.3\right),\left[S_{6},S_{7}\right]\left(0.0\right)\right\}\\ \left\{\left[S_{6},S_{6}\right]\left(0.2\right),\left[S_{6},S_{7}\right]\left(0.8\right),\left[S_{6},S_{6}\right]\left(0.0\right)\right\}\\ \left\{\left[S_{5},S_{7}\right]\left(0.4\right),\left[S_{6},S_{6}\right]\left(0.3\right),\left[S_{5},S_{7}\right]\left(0.3\right)\right\}\\ \left\{\left[S_{5},S_{5}\right]\left(0.3\right),\left[S_{5},S_{6}\right]\left(0.6\right),\left[S_{6},S_{6}\right]\left(0.1\right)\right\}\\ \left\{\left[S_{5},S_{5}\right]\left(0.4\right),\left[S_{5},S_{6}\right]\left(0.6\right),\left[S_{5},S_{5}\right]\left(0.0\right)\right\}\\ \left\{\left[S_{4},S_{4}\right]\left(0.4\right),\left[S_{4},S_{5}\right]\left(0.6\right),\left[S_{4},S_{4}\right]\left(0.0\right)\right\}\\ \left\{\left[S_{4},S_{6}\right]\left(0.3\right),\left[S_{5},S_{5}\right]\left(0.7\right),\left[S_{4},S_{5}\right]\left(0.0\right)\right\}\\ \left\{\left[S_{5},S_{6}\right]\left(0.4\right),\left[S_{5},S_{7}\right]\left(0.6\right),\left[S_{5},S_{6}\right]\left(0.0\right)\right\}\\ \left\{\left[S_{5},S_{5}\right]\left(0.5\right),\left[S_{5},S_{6}\right]\left(0.5\right),\left[S_{5},S_{5}\right]\left(0.0\right)\right\}\\ \left\{\left[S_{4},S_{5}\right]\left(0.2\right),\left[S_{5},S_{5}\right]\left(0.4\right),\left[S_{5},S_{6}\right]\left(0.4\right)\right\}\\ \left\{\left[S_{4},S_{5}\right]\left(0.1\right),\left[S_{4},S_{6}\right]\left(0.3\right),\left[S_{5},S_{6}\right]\left(0.6\right)\right\}\\ \left\{\left[S_{4},S_{5}\right]\left(0.2\right),\left[S_{5},S_{5}\right]\left(0.4\right),\left[S_{5},S_{6}\right]\left(0.4\right)\right\}\\ \left\{\left[S_{4},S_{5}\right]\left(0.2\right),\left[S_{5},S_{6}\right]\left(0.8\right),\left[S_{4},S_{5}\right]\left(0.0\right)\right\}\\ \left\{\left[S_{5},S_{6}\right]\left(0.2\right),\left[S_{6},S_{6}\right]\left(0.4\right),\left[S_{6},S_{7}\right]\left(0.4\right)\right\}\\ \left\{\left[S_{4},S_{6}\right]\left(0.2\right),\left[S_{5},S_{5}\right]\left(0.5\right),\left[S_{5},S_{7}\right]\left(0.3\right)\right\}\\ \left\{\left[S_{5},S_{6}\right]\left(0.2\right),\left[S_{6},S_{7}\right]\left(0.8\right),\left[S_{5},S_{6}\right]\left(0.0\right)\right\}\\ \left\{\left[S_{5},S_{6}\right]\left(0.3\right),\left[S_{6},S_{6}\right]\left(0.3\right),\left[S_{6},S_{7}\right]\left(0.4\right)\right\}\\ \left\{\left[S_{5},S_{7}\right]\left(0.4\right),\left[S_{6},S_{6}\right]\left(0.6\right),\left[S_{5},S_{6}\right]\left(0.0\right)\right\} \end{array}\right]$

**Table 6:** Negative ideal solutions for probabilistic uncertain languages.


$X^{-}=\left[\begin{array}{c} \left\{\left[S_{3},S_{4}\right]\left(0.4\right),\left[S_{4},S_{5}\right]\left(0.3\right),\left[S_{4},S_{5}\right]\left(0.3\right)\right\}\\ \left\{\left[S_{3},S_{5}\right]\left(0.4\right),\left[S_{4},S_{4}\right]\left(0.6\right),\left[S_{3},S_{1}\right]\left(0.0\right)\right\}\\ \left\{\left[S_{5},S_{5}\right]\left(0.5\right),\left[S_{5},S_{6}\right]\left(0.5\right),\left[S_{5},S_{5}\right]\left(0.0\right)\right\}\\ \left\{\left[S_{5},S_{6}\right]\left(1.0\right),\left[S_{5},S_{6}\right]\left(0.0\right),\left[S_{5},S_{6}\right]\left(0.0\right)\right\}\\ \left\{\left[S_{5},S_{6}\right]\left(0.4\right),\left[S_{5},S_{7}\right]\left(0.5\right),\left[S_{6},S_{6}\right]\left(0.1\right)\right\}\\ \left\{\left[S_{5},S_{5}\right]\left(0.6\right),\left[S_{5},S_{6}\right]\left(0.4\right),\left[S_{5},S_{5}\right]\left(0.0\right)\right\}\\ \left\{\left[S_{5},S_{5}\right]\left(0.4\right),\left[S_{5},S_{6}\right]\left(0.4\right),\left[S_{5},S_{7}\right]\left(0.2\right)\right\}\\ \left\{\left[S_{4},S_{5}\right]\left(0.4\right),\left[S_{4},S_{6}\right]\left(0.3\right),\left[S_{4},S_{7}\right]\left(0.3\right)\right\}\\ \left\{\left[S_{4},S_{5}\right]\left(0.4\right),\left[S_{4},S_{4}\right]\left(0.6\right),\left[S_{4},S_{5}\right]\left(0.0\right)\right\}\\ \left\{\left[S_{4},S_{5}\right]\left(0.8\right),\left[S_{5},S_{5}\right]\left(0.2\right),\left[S_{4},S_{5}\right]\left(0.0\right)\right\}\\ \left\{\left[S_{4},S_{5}\right]\left(1.0\right),\left[S_{4},S_{5}\right]\left(0.0\right),\left[S_{4},S_{5}\right]\left(0.0\right)\right\}\\ \left\{\left[S_{4},S_{4}\right]\left(0.4\right),\left[S_{4},S_{5}\right]\left(0.6\right),\left[S_{4},S_{4}\right]\left(0.0\right)\right\}\\ \left\{\left[S_{4},S_{6}\right]\left(0.3\right),\left[S_{5},S_{5}\right]\left(0.7\right),\left[S_{4},S_{5}\right]\left(0.0\right)\right\}\\ \left\{\left[S_{4},S_{5}\right]\left(0.6\right),\left[S_{4},S_{6}\right]\left(0.3\right),\left[S_{5},S_{5}\right]\left(0.1\right)\right\}\\ \left\{\left[S_{4},S_{6}\right]\left(0.6\right),\left[S_{5},S_{5}\right]\left(0.4\right),\left[S_{4},S_{6}\right]\left(0.0\right)\right\}\\ \left\{\left[S_{4},S_{5}\right]\left(0.3\right),\left[S_{4},S_{6}\right]\left(0.3\right),\left[S_{5},S_{5}\right]\left(0.4\right)\right\}\\ \left\{\left[S_{4},S_{6}\right]\left(0.5\right),\left[S_{5},S_{5}\right]\left(0.3\right),\left[S_{5},S_{6}\right]\left(0.2\right)\right\}\\ \left\{\left[S_{4},S_{5}\right]\left(0.3\right),\left[S_{5},S_{5}\right]\left(0.7\right),\left[S_{4},S_{5}\right]\left(0.0\right)\right\}\\ \left\{\left[S_{4},S_{6}\right]\left(0.6\right),\left[S_{5},S_{6}\right]\left(0.4\right),\left[S_{4},S_{6}\right]\left(0.0\right)\right\}\\ \left\{\left[S_{4},S_{5}\right]\left(0.5\right),\left[S_{5},S_{5}\right]\left(0.5\right),\left[S_{4},S_{5}\right]\left(0.0\right)\right\}\\ \left\{\left[S_{5},S_{5}\right]\left(0.3\right),\left[S_{5},S_{6}\right]\left(0.6\right),\left[S_{5},S_{7}\right]\left(0.1\right)\right\}\\ \left\{\left[S_{5},S_{6}\right]\left(1.0\right),\left[S_{5},S_{6}\right]\left(0.0\right),\left[S_{5},S_{6}\right]\left(0.0\right)\right\}\\ \left\{\left[S_{5},S_{5}\right]\left(0.4\right),\left[S_{5},S_{6}\right]\left(0.3\right),\left[S_{6},S_{6}\right]\left(0.3\right)\right\} \end{array}\right]$

**Table 7:** Maximum group utility value and maximum individual regret value.

	Maximum group utility value	Maximum individual regret value
*X*_1_	0.48	0.07
*X*_2_	0.41	0.06
*X*_3_	0.65	0.08
*X*_4_	0.56	0.09

**Table 8:** Compromise values under each decision coefficient.

Decision-making mechanism		*X*_1_	*X*_2_	*X*_3_	*X*_4_
Strengthen the mechanism of individual regret	*v*=0.25	0.35	0.05	0.94	0.90
Balance mechanism	*v*=0.5	0.26	0.01	0.96	0.76
Strengthen group utility mechanism	*v*=0.75	0.12	0.01	0.98	0.70

**Table 9:** Sorting results under each decision coefficient.

Decision-making mechanism		Sorting result
Strengthen the mechanism of individual regret	*v*=0.25	*x*_2_≻*x*_1_≻*x*_3_≻*x*_4_
Balance mechanism	*v*=0.5	*x*_2_≻*x*_1_≻*x*_4_≻*x*_3_
Strengthen group utility mechanism	*v*=0.75	*x*_2_≻*x*_1_≻*x*_4_≻*x*_3_

## Data Availability

The datasets used and/or analyzed during the current study are available from the corresponding author on reasonable request.
